# Resveratrol Prevents GLUT3 Up-Regulation Induced by Middle Cerebral Artery Occlusion

**DOI:** 10.3390/brainsci10090651

**Published:** 2020-09-20

**Authors:** Germán Fernando Gutiérrez Aguilar, Iván Alquisiras-Burgos, Javier Franco-Pérez, Narayana Pineda-Ramírez, Alma Ortiz-Plata, Ismael Torres, José Pedraza-Chaverri, Penélope Aguilera

**Affiliations:** 1 Laboratorio de Patología Vascular Cerebral, Instituto Nacional de Neurología y Neurocirugía “Manuel Velasco Suárez”, Insurgentes Sur #3877, Mexico City 14269, Mexico; gutierrezref@gmail.com (G.F.G.A.); burgos_inc@hotmail.com (I.A.-B.); narayana_pinedar@yahoo.com.mx (N.P.-R.); 2 Laboratorio de Formación Reticular, Instituto Nacional de Neurología y Neurocirugía “Manuel Velasco Suárez”, Insurgentes Sur #3877, Mexico City 14269, Mexico; jfranco@innn.edu.mx; 3 Laboratorio de Neuropatología Experimental, Instituto Nacional de Neurología y Neurocirugía “Manuel Velasco Suárez”, Insurgentes Sur #3877, Mexico City 14269, Mexico; aortizplata@yahoo.com.mx; 4 Unidad del Bioterio, Facultad de Medicina, Universidad Nacional Autónoma de México, Mexico City 04510, Mexico; ismael.torres10@hotmail.com; 5 Departamento de Biología, Facultad de Química, Universidad Nacional Autónoma de México, Mexico City 04510, Mexico; pedraza@unam.mx

**Keywords:** GLUT3, cerebral ischemia, MCAO, resveratrol, astrocytes, AMPK

## Abstract

Glucose transporter (GLUT)3 up-regulation is an adaptive response activated to prevent cellular damage when brain metabolic energy is reduced. Resveratrol is a natural polyphenol with anti-oxidant and anti-inflammatory features that protects neurons against damage induced in cerebral ischemia. Since transcription factors sensitive to oxidative stress and inflammation modulate GLUT3 expression, the purpose of this work was to assess the effect of resveratrol on GLUT3 expression levels after ischemia. Male Wistar rats were subjected to 2 h of middle cerebral artery occlusion (MCAO) followed by different times of reperfusion. Resveratrol (1.9 mg/kg; i. p.) was administered at the onset of the restoration of the blood flow. Quantitative-PCR and Western blot showed that MCAO provoked a substantial increase in GLUT3 expression in the ipsilateral side to the lesion of the cerebral cortex. Immunofluorescence assays indicated that GLUT3 levels were upregulated in astrocytes. Additionally, an important increase in GLUT3 occurred in other cellular types (e.g., damaged neurons, microglia, or infiltrated macrophages). Immunodetection of the microtubule-associated protein 2 (MAP2) showed that MCAO induced severe damage to the neuronal population. However, the administration of resveratrol at the time of reperfusion resulted in injury reduction. Resveratrol also prevented the MCAO-induced increase of GLUT3 expression. In conclusion, resveratrol protects neurons from damage induced by ischemia and prevents GLUT3 upregulation in the damaged brain that might depend on AMPK activation.

## 1. Introduction

Cerebral ischemia occurs when the blood flow in an important cerebral artery is interrupted, depriving the tissue of oxygen and glucose. Consequently, the induction of an irreversible cascade of events, such as excitotoxicity, oxidative stress, apoptosis, and inflammation, provokes neuronal damage. Paradoxically, restoring blood flow (reperfusion) increases reactive oxygen species (ROS) production [1,2]. Oxidative stress stimulates the generation of inflammatory mediators and inflammation that in turn generates ROS. Therefore, it is considered that the interactions between oxidative stress and inflammatory pathways involve positive feedback mechanisms [3].

Accordingly, the use of antioxidants has been recommended as a protective therapy for stroke [4,5,6]. Resveratrol is a stilbene with neuroprotective properties proved in diverse experimental models of neurological diseases including cerebral ischemia [5,7]. Resveratrol’s mechanism of protection is principally associated with its antioxidant capacity, which prevents direct damage to biomolecules [8]. Furthermore, resveratrol directly interacts with proteins, triggering cell signaling pathways that activate anti-oxidant, anti-apoptotic, and anti-inflammatory processes [9,10,11].

Interestingly, ROS increases inflammation by promoting certain stress-activated kinases that stimulate transcription factors such as the nuclear factor kappa B (NF-κB) and the activator protein 1 (AP-1) to induce the expression of pro-inflammatory cytokines [3], as well as the expression of genes involved in controlling the transport of glucose [12,13]. Since the adjustment in glucose transport has been attributed to the neuronal metabolic demand during the post-ischemic period, it is important to understand how the glucose transporters function is regulated [14].

The facilitative glucose transporters (GLUT) are key proteins involved in cellular metabolism because they incorporate glucose to the cerebral parenchyma [15]. There are fourteen members of the GLUT family encoded by the Slc2 genes, the expression of which is regulated during stress conditions [16]. GLUT1 and GLUT3 are highly expressed in the brain and have an essential role in cerebral glucose metabolism [17,18]. GLUT1 is principally expressed in astrocytes, while GLUT3 is known as the neuronal transporter par excellence with a higher affinity for glucose compared to other transporters in the brain [19,20].

Interestingly, GLUT3 expression is up-regulated in the immature and adult brain after global and focal ischemia [14,21,22,23]. Although signaling that activates GLUTs synthesis is unknown, evidence supports that astrocytes are involved in the response. In cultured astrocytes, the oxygen and glucose deprivation (OGD) induces an increase in GLUT3 expression which is mediated by the NF-κB [24]. Conversely, glutamate-mediated excitotoxicity increases glucose transport through trafficking GLUT3 to the neuronal surface [25]. Remarkably, reactive astrocytes, neurons, and microglia secrete cytokines that modify the metabolic phenotype of astrocytes [26,27,28]. In particular, pro-inflammatory cytokines increase glucose consumption and decrease the astrocytic glycogen stores. Unlike astrocytes, neurons are unresponsive to the metabolic effects of cytokines [28]. Therefore, it is probable that the inflammatory process activates a signaling pathway in astrocytes to overcome the energetic challenge induced by ischemia.

Since it has been described that resveratrol’s anti-oxidant and anti-inflammatory properties are associated with protection in ischemia, we hypothesized that resveratrol treatment should not affect GLUT3 up-regulation induced in astrocytes after cerebral ischemia. We confirmed that resveratrol has a protective effect, and intriguingly, our results also indicated that resveratrol significantly diminishes post-ischemic rise in GLUT3 expression at the mRNA and protein level. Treatment prevented GLUT3 up-regulation in astrocytes which might depend on AMPK activation. However, the tremendous rise in GLUT3 expression induced by ischemia was observed in a different type of cell. Since a significant loss of the microtubule-associated protein 2 (MAP2) level, which is considered as indicative of neuronal death, was also observed, we were not able to evaluate the participation of neurons in the increase of GLUT3 expression and consequently, the effect of resveratrol in its prevention. As the presented data are based on a single time of evaluation (24 h of reperfusion), future studies are needed to analyze the involvement of neurons and other types of cells from the very early period after ischemia onset.

## 2. Materials and Methods

### 2.1. Animals

The use of animals was carried out following the protocol No. 23/12 approved by the Institutional Committee for the Care and Use of Animals of the National Institute of Neurology and Neurosurgery “Manuel Velasco Suárez”, under NOM-062-200 and the NIH for the Care and Use of Laboratory Animals. Likewise, the protocol for the use of animals in biomedical research is compatible with the Declaration of the Helsinki World Medical Association. All surgical procedures were performed aseptically, avoiding their suffering as much as possible.

### 2.2. Resveratrol Treatment

An intravenous dose administration was chosen due to low resveratrol bioavailability to allow a greater amount of resveratrol to reach the tissue in its active form at the onset of reperfusion. This dose induces neuroprotection in a similar range than other studies do [7,29,30]. The maximum soluble concentration of resveratrol in 100 µL of the vehicle was used: 1.9 mg resveratrol/kg (R5010, Sigma-Aldrich, St. Louis, MO, USA) diluted in ethanol. Ethanol was prepared at 132 mg/kg of body weight. Resveratrol was administered to animals at the onset of reperfusion by intravenous via (tail vein). For cultures, resveratrol was dissolved in ethanol (0.01%) at a final concentration of 40 μM. Cells were treated at the onset of recovery.

### 2.3. Model of Induction of Transitory Focal Cerebral Ischemia in the Rat

Occlusion of the middle cerebral artery (MCAO) described by Longa et al. [31] was used to induce focal cerebral ischemia. Briefly, male Wistar rats (280–350 g) were anesthetized with 2.5% isoflurane (PiSA, Guadalajara, JAL, Mexico), maintaining oxygen 2% and temperature at 37 °C. The surgery consisted of obstructing the cerebral blood flow to the middle cerebral artery with an intraluminal suture (nylon 3-0) introduced by the left internal carotid artery. After 2 h, animals were anesthetized again and the suture was removed to restore the blood flow. Reperfusion was allowed for different times according to the experiment from 1 to 24 h, and then, animals were sacrificed. The control group underwent the same surgical procedure as the group with MCAO without the insertion of the suture (sham). Physiological parameters were monitored throughout the procedure and animals were maintained at 37 °C after surgery until were completely recovery from anesthesia.

### 2.4. Infarct Area Identification with 2,3,5-Triphenyl Tetrazolium (TTC)

The TTC staining was used to identify the cerebral region damaged by ischemia. Coronal slices of 2.5 mm thick were incubated in 2% TTC solution in PBS (30 min) at 37 °C in the darkness. Subsequently, slices were incubated with 4% paraformaldehyde for 15 min before being photographed. The infarct volume was calculated by measuring the volume of infarct in the slice with respect to the total volume of the slice. Analysis of the images was performed with the ImageJ software 1.8.1 [32].

### 2.5. Ribonucleic Acid (RNA) Extraction

TRIzol^®^ (ThermoFisher Scientific, Waltham, MA, USA) was used to obtain total RNA following manufacturer instructions. One mL Trizol was added to tissue, and combined with 200 μL of chloroform. After 15 min, the mixture was centrifuged (12,000× *g*) for 15 min at 4 °C. Then, the superior phase was mixed with 500 μL of isopropanol. After 10 min at room temperature, the solution was centrifuged (12,000× *g*) for 10 min at 4 °C. Then, the pellet was washed with 75% ethanol and centrifuged (7500× *g*) for 5 min. Lastly, the supernatant was discarded, and the pellet was allowed to desiccate at room temperature. The transparent pill was resuspended in 50 μL of 0.1% diethylpyrocarbonate (DEPC) treated sterile bidistilled water.

### 2.6. Complementary Deoxyribonucleic Acid (cDNA) Synthesis

Five μg of total RNA was used to synthesize the cDNA. The RNA was mixed with hexamers (2.5 μM), reverse transcriptase enzyme buffer (M531A, Promega Corporation, Madison, WI, USA), deoxyribonucleotide triphosphates (dNTPs) (500 μM), RNAsin (20 U), and M-MLV reverse transcriptase (200 U; M1708, Promega Corporation) and DEPC-water. The mixture was incubated 1 h at 37 °C and 5 min at 94 °C. Samples were stored at −20 °C until use.

### 2.7. Quantitative Real-Time Polymerase Chain Reaction (qPCR)

To evaluate the relative level of GLUT3 mRNA expression, the TaqMan^®^FAM probe (Rn01492963_m1, Applied Biosystems, Foster, CA, USA) was employed. The TaqMan^®^VIC probe (Rn01455646_m1, Applied Biosystem) was used to detect the TATA-binding protein and normalize GLUT3 expression. A 7500 Real-Time PCR System (Applied Biosystems) was used to perform the qPCR reactions using Universal PCR Master Mix (4304437, Applied Biosystem). Reactions in triplicate were run under the following conditions: holding step, 95 °C for 10 min, followed by 40 cycles of 92 °C for 15 s and 60 °C for 1 min. The threshold cycle (Ct) was calculated using SDS Software 1.3.1 [33].

### 2.8. Western Blot

To quantify the GLUT3 protein levels, samples were lysed in radioimmunoprecipitation assay buffer (RIPA, 150 mM NaCl, 1% NP40, 1% sodium deoxycholate, 5 mM EDTA, 50 mM HEPES, pH 7.5) supplemented with protease inhibitors (P8340, Sigma-Aldrich). Then, samples were centrifuged (16,000× *g*) for 10 min. The supernatant was recovered, and the protein concentration was calculated by the bicinchoninic acid determination kit (BCA1, Sigma-Aldrich). Electrophoresis was performed on 10% acrylamide gels at constant 110 V for 1 h. Proteins were transferred to polyvinylidene fluoride (PVDF) membranes (162-0115, Millipore, Burlington, MA, USA) during 1 h at 100 V at 4 °C. After, membranes were blocked 1 h with 5% low-fat milk in Tris-buffered saline-Tween (TBS-T) (10 mM Tris Base, 200 mM NaCl, 0.1% Tween 20, pH 7.5). Then, membranes were incubated with antibody anti GLUT3 (1:3000, sc-30107, Santa Cruz Biotechnology, Dallas, TX, USA) overnight at 4 °C, followed by 4 washes of TBS-T (5 mL/10 min) before being incubated with the antibody anti-rabbit IgG conjugated with horseradish peroxidase (1:5000; 115-035-144, Jackson ImmunoResearch, West Grove, PA, USA) for 2 h at room temperature, followed by washes. Signal was detected by chemiluminescence (WBLUF0100, Millipore) using the imaging system Fusion Solo S (Vilber Lourmat, Collégien, France). After that, striping buffer (15 g glycine, 1 g sodium dodecyl sulfate (SDS), 10 mL Tween 20, pH 2.2) was added to the PVDF membrane for 20 min, washed with TBS-T, and blocked again to incubated with α-tubulin (1:3000; T9026, Sigma-Aldrich), the protein used to normalize protein concentration, followed by the antibody anti-mouse IgG conjugated with horseradish peroxidase (1:10,000; 115-035-003, Jackson ImmunoResearch).

### 2.9. Immunofluorescence

Rats were anesthetized intraperitoneally with 100 mg/kg of pentobarbital (PiSA), and then perfused transcardially with 4% paraformaldehyde in phosphate buffered saline (PBS). The brains were fixed in 4% paraformaldehyde (24 h), and successively placed in augmented concentrations of sucrose (10%, 20%, and 30%) for three days at 4 °C. Coronal sections of 10 μm were obtained (freezing microtome Sartorius-Werke, model 27, Gottingen, Germany) and stored at −20 °C in 30% ethylene glycol and 20% glycerol in PBS, pH 7.4, until use. Coronal sections were permeabilized with 0.1% Triton X-100 in PBS (30 min) and blocked with 10% goat serum in PBS (60 min). Then, antibodies anti Microtubule-Associated Protein 2 (1:750; MAP-2, AB5392, Abcam, Cambridge, UK), anti-Glial Fibrillary Acid Protein (1:750; GFAP, Z0334, Dako, Carpinteria, CA, USA), and anti GLUT3 (1:500; sc-30107, Santa Cruz) were incubated in 1% bovine serum albumin in PBS overnight at 4 °C. Then, sections were washed and incubated with Alexa Fluor^®^ 594-conjugated anti-chicken IgG (703-585-155), Alexa Fluor^®^ 594-conjugated anti-rabbit IgG (711-585-152) or DyLight™ 488-conjugated anti-mouse IgG (715-485-150) from Jackson ImmunoResearch Laboratories Inc or Alexa Fluor^®^488-conjugated anti-rabbit IgG (1500-73; Abcam) as required. To identify nuclei, coronal sections were incubated with 1 µg/mL 4′, 6-diamidino-2-phenylindole (DAPI) to detect nuclei (Sigma-Aldrich) (15 min) and mounted with Mowiol (4.8% Mowiol 4.88, 0.1% p-phenylenediamine, 12% glycerol, 0.02% NaN_3_, and 0.2 M Tris-HCl). The sections were obtained from Bregma 1.0 to −0.4 mm and images were taken in the ipsilateral region of the cerebral cortex. Four images were acquired in each slice (*n* = 3) using 20× dry objective lenses in an inverted microscope Olympus 1 × 71 (Olympus Corporation of the Americas, Center Valley, PA, USA). Image J software 1.8.0 was used to perform the imaging analysis [32]. Colocalization analysis was performed as follows: 1) Channels were separated with the channel split function; 2) Colocalization of the green (GLUT3) and red (GFAP or MAP2) channels was analyzed using the function for colocalization thresholds. Colocalization was reported as “R” total of MAP2 or GFAP/GLUT3 corresponding to Pearson’s correlation coefficient. The coefficient ranges from −1 to 1, a result near +1 means perfect correlation, 0 indicates no correlation, and −1 for perfect anti-correlation.

### 2.10. Primary Culture of Neurons and Astrocytes from the Cerebral Cortex

Embryos (E17–18) were removed from the yolk sac and placed in cold Hank’s Buffer Saline Solution (0.14 mM NaCl, 5.33 mM KCl, 0.44 mM KH_2_PO_4_, 5.56 mM glucose, and 0.34 mM Na_2_HPO_4_). The brain was removed and transferred to cold a DMEM™ culture medium (D1152-1L, Thermo Scientific). Cerebral cortices were dissected and transferred to Neurobasal™ medium (21103049, Thermo Scientific) supplemented with B27™ 1X (17504-044, Thermo Scientific) and GlutaMAX™ 1X (35050-061, ThermoFisher Scientific). Then, tissue was enzymatically disintegrated with 3 mL of a trypsin solution for 5 min at 37 °C, and the reaction was inhibited with 1 mL of fetal bovine serum (FBS; S1810, BIOWEST, Nuaillé, France). The homogenous solution was passed through a 70-μm filter, and seeded at a density of 25,000 cells/cm^2^. After three days, 50% of the culture medium was replaced (it was not supplemented with cytosine arabinoside to allow the growth of astrocytes). Cells were maintained at 37 °C, 21% O_2_, and 5% CO_2_. Experiments were carried out after 7 days in vitro (DIV). The presence of neurons was established by immunofluorescence, using the specific neuronal tag, the MAP-2 and astrocytes by the presence of the GFAP. Hoechst 3342 (Sigma Aldrich) was used to detect nuclei.

To induce excitotoxicity, cultures were treated with L-glutamate (100 µM) and glycine (10 µM) for 10 min. Cultures were divided into: CT, cells to which the culture medium was changed by Krebs–Henseleit solution (KHB) solution followed by recovery; GLU, cells with induced excitotoxicity followed by recovery; GLU + RSV, cells exposed to excitotoxicity plus resveratrol (40 μM).

### 2.11. Immunofluorescence in Cultures

Cells seeded on glass coverslips in 24-well plates were fixed with formaldehyde (0.5% in PBS, 10 min), permeabilized with cooled methanol (−70 °C, 1 min), washed with ice-cooled PBS (5 min), and blocked with bovine serum albumin (5% in PBS, 1 h, at room temperature). Subsequently, cells were incubated with Hoechst 33,342 (10 μg/mL) and the antibody anti-phospho-Thr 172-adenosine monophosphate (AMP)-activated protein kinase (AMPK) α (2531, Cell Signaling Technology, Danvers, MA, USA) at 4 °C, overnight. Additionally, the anti-MAP-2 antibody was used to identify neurons. After incubation, cells were washed with ice-cooled PBS (3 times, 10 min) and then incubated with the secondary antibodies Alexa Fluor^®^ 594-conjugated anti-chicken IgG or DyLight™ 488-conjugated anti-mouse IgG (2 h, at 37 °C). Followed by washes with ice-cooled PBS (3 times, 10 min). The coverslips were mounted with Mowiol. Fluorescence was detected with an inverted microscope Olympus model 1 × 71 using a 20× dry objective.

### 2.12. Statistical Analysis

Statistical data were acquired from at least 3 independent experiments. Data were presented as the mean ± standard deviation. The analysis of variance of one way (ANOVA) followed by Tukey was performed using the GraphPad Prism 5 software (Inc. San Diego, CA, USA).

## 3. Results

### 3.1. Resveratrol Reduces the Damage Induced by the MCAO

We measured the infarct area induced by 2 h of MCAO with the TTC staining (Figure 1A,B) and found that resveratrol has a protective effect as has previously demonstrated [29]. We also performed an immunofluorescence assay to detect MAP2 expression because its loss reflects cytoskeletal breakdown and represents a sensitive marker of ischemic damage [34]. We observed an evident reduction in the MAP2 signal in the MCAO + VH (vehicle) group, an alteration that represents a loss of axons integrity. When animals were treated with resveratrol, integrity of the fibers was conserved (Figure 1C,D). These results evidence that resveratrol avoided damage to the tissue and suggested the preservation of neuronal viability.

### 3.2. The GLUT3 mRNA Up-Regulation Induced by MCAO is Prevented by Resveratrol Treatment

There are works showing that GLUT3 mRNA level is modified in different experimental models of ischemia [21]. We found that ischemia increased the level of expression of GLUT3 in the cerebral cortex at the ipsilateral side to the lesion. The highest level of expression was detected very early after reperfusion (2.5 ± 0.61-fold). Subsequently, GLUT3 mRNA returned to basal levels and was maintained from 3 to 8 h of reperfusion (Figure 2A).

Because GLUT3 expression depends on transcription factors known to be regulated by resveratrol, we assessed its effect on the up-regulated GLUT3 mRNA levels induced by the MCAO. Experiments showed that resveratrol prevents the rise in the mRNA induced by 2 h of MCAO and 1 h of reperfusion (Figure 2B).

### 3.3. Resveratrol Prevents the Increase in the GLUT3 Protein Levels Induced by Ischemia and Reperfusion

The up-regulation in the mRNA levels is normally accompanied by a subsequent increase in protein concentration. Therefore, Western blot analysis was performed to corroborate that the effect of resveratrol on the GLUT3 mRNA levels correlated with GLUT3 protein expression. We found that 2 h of ischemia followed by 24 h of reperfusion stimulated a significant increase in GLUT3 protein level (3.4 ± 0.3-fold; Figure 3A,B). Consistent with the results found at the mRNA level, resveratrol administered at the onset of reperfusion also prevented the increase in the level of GLUT3 protein induced by the MCAO (Figure 3A,B).

### 3.4. GLUT3 Over Expression Induced after MCAO Does Not Overlap with MAP2 Signal

Immunofluorescence analysis was performed to assess whether MCAO and resveratrol alters expression of GLUT3 in a specific cell type. First, we confirm that GLUT3 is a protein with a high expression in neurons of the control brain while astrocytes are expressed at very low levels (Figure 4).

Then, we evaluated the effect of resveratrol in the MCAO groups. Because the rise induced by ischemia in the GLUT3 expression was huge, the intensity of the signal obtained in the microscope was downgraded in control groups to allow a proper quantification in Figure 5A,B (1.74 ± 0.69). After the insult, the increment on GLUT3 expression was significant, reaching 9.8 ± 2.4. As previously observed by Western blot, the increase induced by MCAO was prevented with resveratrol treatment (Figure 5A,B).

After, the MAP2 level was detected to evaluate the abundance of GLUT3 in neurons. When colocalization of both proteins was quantified, we found that the GLUT3/MAP2 ratio did not increase after ischemia (Figure 6). However, MAP2 is a sensitive marker to damage, therefore the colocalization could be underestimated.

### 3.5. MCAO Induces GLUT3 Up-Regulation in Astrocytes

Given the essential role of astrocytes in the transference of substrates to neurons [35], we next evaluated the expression of GLUT3 in cells positive to the astrocyte-specific mark GFAP. GFAP is a cytoskeleton protein, the levels of expression of which have been associated with inflammatory response to damage [36]. As previously showed, GLUT3 was up-regulated. Interestingly, GLUT3 overlapping with GFAP was significantly increased with MCAO and resveratrol prevented both the up-regulation and colocalization of GLUT3 with GFAP (Figure 7A,B).

### 3.6. Resveratrol Induces Phosphorylation of AMPK

It is known that AMPK directly activates SIRT [37]. SIRT1 inhibits the transcriptional activity of p65-NF-κB, an important regulator of GLUT3 expression [24]. Therefore, we decided to evaluate the effect of resveratrol on the level of p-AMPK to identify a possible pathway of p65-NF-κB inactivation. We used mixed cultures of neurons and astrocytes exposed to glutamate-induced excitotoxicity, a model of ischemic stroke (Figure 8A). We observed that both excitotoxicity and resveratrol increased p-AMPK signal (Figure 8B,D). The increase in p-AMPK was found in neurons and also in non-MAP2 positive cells (i.e., astrocytes) (Figure 8C).

## 4. Discussion

The obstruction of blood flow during cerebral ischemia results in a critical depletion of cell energy. Consequently, the rapid restoration of nutrient supply is essential to maintain neuronal functions. Evidence suggests that cells integrating the neurovascular unit respond by up-regulating the expression of glucose transporters [21]. This response has been associated with a reduction of brain lesions in neurodegenerative diseases and traumatic brain injury [38,39].

In the present work, we observed that ischemia induced a substantial up-regulation of GLUT3 in the rat brain subjected to MCAO. We found an increase in GLUT3 expression within GFAP positive cells. Interestingly, in the healthy brain, GLUT3 gene expression is mainly limited to neurons [40,41]. Even so, in glioma cells, GLUT3 is the predominant glucose transporter [42]. Likewise, increased expression of GLUT3 occurs in astrocytes located in the center of chronic active lesions of multiple sclerosis disease, whereas axons showed a reduced expression [39]. Also, after 5 min of transient forebrain ischemia, a strong GLUT3 immunoreactivity is found in astrocytes in the hippocampus but not in differentiated neuroblasts [43]. Moreover, the specificity protein (SP), the hypoxia inducible factor-1α, and NF-κB modulate the expression of GLUT3 in astrocytes [24,42,44]. Therefore, the increase in GLUT3 synthesis observed after cerebral ischemia proposes the participation of astrocytes in the rescue of neurons to ensure sufficient nutrient transport under stress conditions and suggest the activation of the adaptative response to modulate glucose level [36].

We also found that MCAO induces an increase in GLUT3 expression in cells not expressing GFAP. Although neurons can detect glucose levels and adjust their transport, it is well known that fluctuating glucose levels modify the mitochondrial activity, activate apoptosis, and induce pro-inflammatory factors [45,46,47]. Therefore, the regulation of GLUT3 expression in neurons could represent a manner in which resveratrol induces protection. We used MAP2 as a neuronal marker to identify co-localization with GLUT3. However, MAP2 is a sensitive marker that begins to disappear as soon as 1 h after MCAO onset [48]. Because we performed the quantification 24 h after ischemia, the MAP2 signal was negligible and gave us little information. Therefore, the observed increased expression of GLUT3 could have occurred in neurons in which MAP2 was no longer detected because of the injury. Additionally, damage to the blood–brain barrier during ischemia could allow the infiltration of immune cells, which express high GLUT3 levels, and also in activated microglia [49,50,51,52,53,54]. Therefore, it will be essential to characterize the expression of GLUT3 in neurons at earlier times of reperfusion and in other types of cells.

The protective effect of resveratrol has been tested in many experimental models, where ROS provokes damage [52]. Previously, we demonstrated that resveratrol administered at the beginning of reperfusion reduces tissue damage and the neurological deficit induced by MCAO [29]. Here, we found that ischemia reduced the infarct area and the MAP2 level of expression, this effect represents an alteration in the microtubule structure of the cytoskeleton and signifies a reduction in the number of surviving neurons [34,48,53]. Importantly, the cytoskeleton alteration observed in neurons was reduced with resveratrol treatment. This situation might be associated with the presence of neurons that maintain viability and is in consensus to the resveratrol’s protective effect.

When we investigated the effect of resveratrol in the up-regulation of GLUT3 expression induced by MCAO, we found that resveratrol significantly prevented it. Resveratrol modulates signaling pathways that depend on the redox state of the cell. For instance, SP, a transcription factor sensitive to oxidative stress has a relevant participation in GLUT3 mRNA synthesis [42,54]. The DNA binding activity of SP is blocked by resveratrol treatment after MCAO [29]. Consequently, it is possible that resveratrol blocks the SP binding to the promoter region of the GLUT3 gene, inhibiting its overexpression after MCAO.

In the current study, we found that resveratrol induces the phosphorylation of AMPK in mixed cultures of neurons and astrocytes subjected to excitotoxicity. It is relevant because glutamate excitotoxicity, cytokines, and high glucose induce NF-κB activation, a transcription factor involved in GLUT3 up-regulation in astrocytes [24,55,56]. Interestingly, resveratrol reverses high-glucose-induced inflammation by activating the AMPK/SIRT1/NF-κB pathway [55,57,58] and inhibits the transactivation of p65-NF-κB [59]. Additionally, resveratrol induces AMPK activation at early times of reperfusion in the in vivo model of MCAO, and compound C, an AMPK inhibitor prevents its protective effects [30]. Thus, it is also possible that resveratrol, through the activation of AMPK, down-regulates the GLUT3 expression induced after MCAO, which could occur in both neurons and astrocytes.

## 5. Conclusions

Resveratrol treatment resulted in a decrease in ischemic-induced damaged and also prevented the increase in GLUT3 expression. Our results indicated that astrocytes were partially responsible for the over-expression of GLUT3 after 2 h of MCAO and 24 h of reperfusion, and neurons could be also implicated at earlier times. It is known that GLUT3 up-regulation has a protective role against cerebral damage. However, we cannot exclude the possibility that the effect of resveratrol could be associated with an endogenous response that prevents glucose-induced toxicity in neurons and activates a compensatory mechanism in astrocytes. Nonetheless, our current study is initial, and additional research is required to better understand of the process.

## Figures and Tables

**Figure 1:** Resveratrol protects the brain from damage induced by ischemia. Rats were subjected to middle cerebral artery occlusion (MCAO) during 2 h followed by restoration of blood flow (reperfusion) for 24 h. Control animals (CT) were subjected to simulated MCAO. At the onset of reperfusion, rats received either vehicle, ethanol 50% (+VH) or resveratrol at 1.9 mg/kg, body weight (+RSV). Immunofluorescence was used to detect microtubule-associated protein 2 (MAP2) protein expression in neurons. 4′, 6-diamidino-2-phenylindole (DAPI) was used to detect nuclei. (**A**) Infarct area detected by 2,3,5-triphenyl tetrazolium (TTC) staining. (**B**) Quantification of the infarcted area. (**C**) Images show in red the signal associated to MAP2 and blue the nuclei. NEG, Negative control without primary antibody. (**D**) Quantification of MAP2 expression. Fluorescence was reported in % of the signal associated to MAP2 in the region of interest (ROI). Values were expressed as mean ± standard deviation. ANOVA, Tukey, * *p* < 0.05, *** *p* < 0.001.

**Figure 2:** Resveratrol prevents the ischemia induced glucose transporter 3 (GLUT3) mRNA up-regulation in the brain. Rats were subjected to middle cerebral artery occlusion (MCAO) during 2 h followed by restoration of blood flow (reperfusion) for 24 h. Control animals (CT) were subjected to simulated MCAO. At the onset of restoration of blood flow, animals received either vehicle, ethanol 50% (+VH) or resveratrol at 1.9 mg/kg, body weight (+RSV). Relative mRNA expression was measured by quantitative PCR. (**A**) GLUT3 mRNA levels after MCAO and different times of reperfusion. (**B**) The effect of resveratrol on GLUT3 mRNA levels induced after MCAO and 1 h reperfusion. Values of expression were expressed as mean ± standard deviation. ANOVA, Tukey, * *p* < 0.05.

**Figure 3:** Resveratrol prevents glucose transporter 3 (GLUT3) up-regulation induced in the brain after ischemia. Rats were subjected to middle cerebral artery occlusion (MCAO) during 2 h followed by restoration of blood flow (reperfusion) for 24 h. Control animals (CT) were subjected to simulated MCAO. At the onset of restoration of blood flow, animals received either vehicle, ethanol 50% (+VH) or resveratrol at 1.9 mg/kg, body weight (+RSV). (**A**) GLUT3 protein expression measured by immunoblotting. (**B**) Quantification of the effect of resveratrol on GLUT3 protein after cerebral ischemia. Values were expressed as mean ± standard deviation. ANOVA, Tukey, *** *p* < 0.001, **** *p* < 0.0001.

**Figure 4:** Glucose transporter 3 (GLUT3) expression in neurons and astrocytes in the control brain. Brain coronal sections were obtained from control rats and analyzed by immunofluorescence. Images were acquired on a Nikon Ti Eclipse inverted confocal microscope using a 20x objective lenses. (**A**) Nuclei (blue), 4′, 6-diamidino-2-phenylindole (DAPI) was used to detect nuclei, (**B**) GLUT3 (green), (**C**) Neuronal specific protein: the microtubule-associated protein 2 (MAP2, red), (**D**) Astrocyte specific protein: glial fibrillary acid protein (GFAP, violet), (**E**) Low expression of GLUT3 in GFAP positive cells, (**F**) High expression of GLUT3 in MAP2 positive cells, and (**G**) Merge of DAPI, GLUT3, MAP2 and GFAP signal, showing predominant expression of GLUT3 in neurons.

**Figure 5:** Resveratrol prevents glucose transporter 3 (GLUT3) up-regulation induced in the brain after ischemia. Rats were subjected to middle cerebral artery occlusion (MCAO) during 2 h followed by restoration of blood flow (reperfusion) for 24 h. Control animals (CT) were subjected to simulated MCAO. At the onset of restoration of blood flow, animals received either vehicle, ethanol 50% (+VH) or resveratrol at 1.9 mg/kg, body weight (+RSV). (**A**) Immunofluorescence of GLUT3 (green) protein expression. 4′, 6-diamidino-2-phenylindole (DAPI) was used to detect nuclei (blue). (**B**) Quantification of GLUT3 expression. Fluorescence was reported in % of the signal associated with GLUT3 in the region of interest (ROI). Values of ROI were expressed as mean ± standard deviation. ANOVA, Tukey, ** *p* < 0.01, *** *p* < 0.001.

**Figure 6:** Glucose transporter 3 (GLUT3) expression is not increased in neurons after MCAO. Rats were subjected to middle cerebral artery occlusion (MCAO) during 2 h followed by restoration of blood flow (reperfusion) for 24 h. Control animals (CT) were subjected to simulated MCAO. At the onset of restoration of blood flow, animals received either vehicle, ethanol 50% (+VH) or resveratrol at 1.9 mg/kg, body weight (+RSV). Immunofluorescence was used to detect GLUT3 protein expression in neurons. 4′, 6-diamidino-2-phenylindole (DAPI) was used to detect nuclei. (**A**) Representative images show GLUT3 (green), microtubule-associated protein 2 (MAP2) (red), and nuclei (blue). NEG, Negative control without primary antibody. (**B**) Quantification of the fluorescence for GLUT3 expression in cells positive for the neuronal marker MAP2. Fluorescence was reported as R (Pearson’s correlation coefficient) of the signal associated with the colocalization of MAP2 and GLUT3 proteins in the region of interest (ROI). Values were expressed as mean ± standard deviation. ANOVA, Tukey, NS, not significant.

**Figure 7:** Resveratrol prevents the ischemia induced increase in glucose transporter 3 (GLUT3) expression. Rats were subjected to middle cerebral artery occlusion (MCAO) during 2 h followed by restoration of blood flow (reperfusion) for 24 h. Control animals (CT) were subjected to simulated MCAO. At the onset of restoration of blood flow, animals received either vehicle, ethanol 50% (+VH) or resveratrol at 1.9 mg/kg, body weight (+RSV). Immunofluorescence was used to detect GLUT3 protein expression in astrocytes. 4′, 6-diamidino-2-phenylindole (DAPI) was used to detect nuclei. (**A**) Representative images of GLUT3 (green), glial fibrillary acid protein (GFAP) (red), and nuclei (blue). (**B**) Quantification of GLUT3 expression astrocytes. Fluorescence quantification of the astrocyte (cells positive to GFAP) expressing GLUT3. Fluorescence was reported as R (Pearson’s correlation coefficient) of the signal associated with the co-localization of GFAP and GLUT3 proteins in the region of interest (ROI). Values were expressed as mean ± standard deviation. ANOVA, Tukey, * *p* < 0.05, *** *p* < 0.001.

**Figure 8:** Resveratrol increases AMP-activated protein kinase (AMPK) phosphorylation. Primary mixed cultures of neurons and astrocytes of 7–8 days in vitro were stimulated with 100 μM glutamate (GLU) and 10 μM glycine to induce excitotoxicity and allowed to recover for 20 min. Cultures were divided into CT, control; GLU, exposed to excitotoxicity, GLU + RSV, plus resveratrol [40 μM]. Immunofluorescence. Cultures were stained with Hoechst 33,342 (blue) to identify nuclei, anti- microtubule-associated protein 2 (MAP2) followed by Alexa Fluor^®^ 594 (red) to identify neurons, and anti- glial fibrillary acid protein (GFAP) or anti phospho AMPK(p-AMPK) followed by DyLight™ 488 (green) to identify astrocytes or phosphorylate AMPK. (**A**) Detection of the cellular types in the culture. (**B**) Detection of anti phospho AMPK (p-AMPK, green). (**C**) Co-localization of MAP2 and p-AMPK. (**D**) Quantification of the fluorescence for p-AMPK expression. Fluorescence was quantified and reported as “fold” of the intensity of the pixels in a region of interest (ROI). Values of ROI were expressed as mean ± standard deviation. ANOVA, * *p* < 0.05; N.S., not significant.
